# Change in Self-Reported Health Status among Immigrants in the United States: Associations with Measures of Acculturation

**DOI:** 10.1371/journal.pone.0076494

**Published:** 2013-10-01

**Authors:** Sunmin Lee, Allison H. O’Neill, Emily S. Ihara, David H. Chae

**Affiliations:** 1 Department of Epidemiology and Biostatistics, University of Maryland School of Public Health, College Park, Maryland, United States of America; 2 Department of Social Work, George Mason University, Fairfax, Virginia, United States of America; University of California, United States of America

## Abstract

Although acculturation may have positive effects for immigrants, including better socioeconomic profiles and increased occupational opportunities, their health profiles deteriorate with longer duration in the U.S. Prior research indicates that increasing acculturation is associated with some poorer health outcomes among immigrants in the U.S. However, most of these studies have used length of stay or English language proficiency as proxies for acculturation, and have mainly examined self-reported “current” health outcomes. This study advances knowledge on associations between acculturation and health among immigrants by explicitly examining self-reported “change” in health since immigration, in relation to acculturation-related variables. We use data from the New Immigrant Survey (NIS; 2003-2004), a cross-sectional study of legal immigrants to the U.S. In addition to testing more conventionally examined proxies of acculturation (length of stay and English proficiency), we also examine English language use and self-reported change in diet. Multivariable logistic regression analyses on 5,982 participants generally supported previous literature indicating a deleterious impact of acculturation, with increasing duration of stay and greater self-reported change in diet being associated with a poorer change in health since moving to the U.S. Although English language proficiency and use were associated with greater odds of reporting a worse change in health when examined individually, they were non-significant in multivariable models including all acculturation measures. Findings from this study suggest that when taking into account multiple measures of acculturation, language may not necessarily indicate unhealthy assimilation and dietary change may be a pathway leading to declines in immigrant health. Increasing duration in the U.S. may also reflect the adoption of unhealthy behaviors, as well as greater exposure to harmful sources of psychosocial stress including racial and anti-immigrant discrimination. Our study suggests that multiple indicators of acculturation may be useful in examining the effect of acculturation on changes in health among immigrants.

## Introduction

Although immigrants conventionally display improved socioeconomic profiles with increasing duration in the U.S. or through successive generations, the opposite holds true for health outcomes, an effect known as unhealthy assimilation [1,2]. Unhealthy assimilation or deterioration in health status raises questions about the social environmental factors that are associated with the health of immigrants and their descendents. Research has consistently shown an inverse relationship between socioeconomic position and health across various self-reported measures and clinical observations of disease [3-9]. However, immigrants, even those with lower socioeconomic positions, have generally been shown to have better health compared to their native born counterparts at the time of or shortly after immigration [10-13]. The “healthy immigrant effect” refers to the paradox that despite often having worse socioeconomic characteristics, less access to health care services, and experiencing greater linguistic and cultural barriers related to accessing health information, immigrants tend to have better health profiles compared to their native-born counterparts [11,14]. Several studies have shown that this health advantage deteriorates over time and with successive generations in the U.S. [10,15-17] as well as in other countries [18-20].

Researchers have posited two primary explanations for this paradox: selective migration and cultural “buffering.” Selective migration suggests that individuals who are healthier and more resilient may be more likely to migrate; and conversely, that those who are older or become unhealthy may choose to return to their home countries, thus altering the death statistics and health profiles of those remaining [21-25]. The cultural buffering hypothesis suggests that culturally-specific health protective and promotive behavior and contexts are more influential for good health outcomes than conventional risk factors such as low socioeconomic position [1,22,26]. This explanation points to the cultural norms and values of the immigrant group that decrease risky behaviors, provide stronger social and familial support, and encourage better nutrition choices as mechanisms for better health [27-31]. With increased acculturation, however, cultural buffering begins to erode and health deteriorates toward less healthy U.S. norms [11,21,30]. Some researchers argue that these two hypotheses are complementary and that there may be positive health selection which creates healthier profiles for immigrants. However, as immigrants are exposed to various social hazards of the host society, this health advantage declines over time [11,16].

The process of acculturation is complex and multidimensional. Acculturation is most often conceptualized as a process by which an immigrant adopts the language, customs, behaviors, and attitudes of the host culture [32,33]. Once thought to be a unilinear and directional process [34], theoretical work in this area has advanced scholarly thinking to account for the multidimensional ways immigrants interact with their host culture. For example, biculturalism suggests that individuals can be oriented both toward their cultures of origin and the host culture simultaneously [35,36]; economic integration posits that immigrants may integrate economically without culturally assimilating [37]; and structural context models incorporate the role of both socioeconomic factors and psychosocial stress [32,38,39].

Several studies of acculturation and health show that the immigrant health advantage deteriorates over time, which may be attributed to adoption of less healthy American lifestyles, including those around diet, smoking, body mass index, and physical activity [40-46]. In the classic study by Marmot and Syme, men of Japanese ancestry living in the U.S. were shown to have elevated incidence rates of coronary heart disease (CHD) compared to those living in Japan. Furthermore, Japanese Americans most acculturated to Western culture had a prevalence of CHD three to five times higher than those who retained their Japanese traditional culture [2].

There is increasing evidence that greater length of stay in the U.S. is associated with worse health among immigrants. A recent report using the Current Population Survey found that first generation immigrants were less likely to rate their health as poor/fair than third generation and more acculturated immigrants. Longer length of stay in the U.S. was also associated with greater poor/fair self-rated health for Asians and Hispanics [10]. Data from the California Health Interview Survey (CHIS) also revealed that compared to native-born respondents, immigrants reported better health, but this effect diminished with increasing length of stay in the U.S. [47]. Another study using data from the New Immigrant Survey reported that Hispanic immigrants who rated their current health as “worse” than before coming to the U.S. were on average living in the U.S. two years longer compared to those who rated their health as being “better” than before coming to the U.S. [40]. Other studies on Asian and Pacific Islander groups have found evidence for higher risk for health problems associated with increasing duration in the U.S. [11].

Collectively, research findings suggest that increasing length of stay in a new country, often used as a proxy for acculturation, may be associated with declines in health. However, acculturation may be measured using alternative measures, such as changes in diet, and English language use and proficiency. Language of the study interview may be a particularly robust measure of acculturation for Asians. For example, data from the CHIS revealed that foreign-born Asians who interviewed in English more closely resembled U.S.-born Asians on demographic, health status, and health behavior variables compared to foreign-born Asians who interviewed in other languages [48]. Diet has been studied as a component of acculturation in previous literature [49,50]. A review by Perez-Escamilla & Putnik (2007) in the Journal of Nutrition highlights studies that have shown an association between dietary variables (such as consumption of fruits and vegetables) and acculturation [49].

Another study using the New Immigrant Survey suggested that diet may also be a salient marker of acculturation among Hispanics. In this study, Hispanic immigrants who had been in the U.S. longer reported more dietary changes, and that change in diet was associated with higher body mass index [40].

The present study aims to examine how acculturation, measured by length of stay in the U.S., English use and proficiency, and diet change, is associated with change of health status in immigrants using data from the New Immigrant Survey (NIS). A novelty of this study is the use of self-reported “change” in health status, whereas most prior studies have examined only self-reported “current” health status. Although the data for the present study is cross-sectional, inferences regarding the relative decline or improvement of health as a result of immigration are more fully supported. Another strength of the current study is the inclusion of multiple measures of acculturation to take into consideration various aspects of acculturation. Additionally, this study includes participants from diverse immigrant populations, including those from Sub-Saharan Africa, Canada, Asia, South and Central America, and the United Kingdom. We test the following hypotheses:

1 Compared to more recently arrived immigrants, those with longer length of stay in the U.S. are more likely to report worse change in health than before moving to the U.S.; and
2 Immigrants who report higher English proficiency, greater English use, and greater changes in diet will report worse health than before moving to the U.S. compared to those who report less English proficiency and use and fewer changes in diet.

## Materials and Methods

### Ethics Statement

The New Immigrant Survey, the dataset used in this study, has received Institutional Review Board approval from Princeton University Institutional Review Board and all appropriate sources.

### Study participants

The New Immigrant Survey (NIS) is a nationally representative study of legal immigrants to the U.S. Immigrants granted permanent residence from May to November 2003 were sampled using U.S. government electronic administrative records. About 60% of study participants lived in the U.S. less than equal to five years. them tended to be recent Data used for this study were collected from June 2003 to June 2004 [51]. The data are publicly available from the following website: http://nis.princeton.edu/. Interested users can register and download the data.

The survey sample included 8,573 adult immigrants. Circular migrants who moved to the U.S. more than once were excluded from our analyses (n = 608, 7.1%). Also excluded were indirect immigrants, or those who moved from their country of birth to another country, and then subsequently moved to the U.S. (n = 1,185, 13.8%). These two groups of immigrants were excluded from analyses because their experiences of acculturation are likely to be qualitatively different from those who moved directly to the U.S., by having either additional exposure to their countries of origin or having had to adapt to multiple new environments. Additionally, participants with missing data on migration history prior to coming to the U.S. were excluded (n = 141, 1.6%).

One hundred and twenty participants (1.4%) with missing data on self-reported change in health, 24 participants with missing data on year on birth (0.3%), 139 participants with missing data on year of migration (139, 1.6%), and 374 participants with missing data on language variables (4.4%) were also excluded from the current study. The final analytic sample consisted of 5,982 participants (unweighted; 5,991, weighted).

### Measures

#### Length of Stay in the U.S

Length of stay in the U.S. was defined as the year of moving to the U.S. subtracted from the year of interview. Length of stay in the U.S. has been found to be an objective indicator of acculturation, and has been routinely examined in studies of acculturation among immigrants [10,11,52-54]. Length of stay in the U.S. was categorized into the following levels: less than 1 year (referent); 1-5 years; 6-10 years, 11-15 years, and 16 or more years [55].

#### English Proficiency

English proficiency was also examined as a proxy of acculturation, measured using two separate items which asked participants to rate: (1) their English speaking; and (2) their comprehension as “very well”, “well”, “not well”, or “not at all”. In the current study, we constructed a dichotomous variable of “not well or not at all” (referent) vs. “very well or well” for each individual item.

#### English Use

Additional language variables examined in the current study were language spoken at work, language spoken at home, and language spoken with friends. Each of these variables was grouped as “English” (referent) vs. “non-English”.

#### Dietary Change

Dietary change was assessed using a single item measured on a 10-point Liker scale, asking participants to rate the degree to which their diet has changed since moving to the U.S., with 1 = completely different, and 10 = completely the same. Participants were divided into five categories of: completely different (a value of 1); very different (values ranging from 2 to 4); somewhat different (a value of 5); very similar (values ranging from 6 to 9); and completely the same (a value of 10). These categories were constructed based on *a priori* cut-points and the distribution of responses.

#### Change in Health Status

Participants were asked to indicate how their health status has changed when comparing their health now to right before they came to the U.S. Response options included better, about the same, and worse. Responses were dichotomized into those with worse health vs. those with the same or better health (referent).

#### Sociodemographic Factors

Covariates included self-reported measures of: gender; age, calculated by subtracting year of birth from year of interview; years of education, categorized into less than 12 years, 12-16 years, and more than 16 years; marital status, categorized as never married, separated/divorced/ widowed, and married or living with a significant other; and health insurance (any, including private or public sources such as Medicaid, vs. none). Race/ethnicity was categorized into: Hispanic, Non-Hispanic White, Non-Hispanic Black, Asian, and Multiracial/Other. Self-reported health behaviors that were examined were smoking (current, former, or never); and self-reported exercise, categorized as >3 times per week, <3 times per week, or none. Self-reported height and weight were used to calculate body mass index (BMI), and participants were categorized as underweight (

< 18.5 kg/m^2^), normal (18.5-25 kg/m^2^), overweight (25-30 kg/m^2^), and obese (>30 kg/m^2^).

### Data Analysis

Bivariate associations between each of the seven acculturation variables (length of stay in the U.S., English speaking ability, English comprehension, language at home, language at work, language with friends, and change in diet) and self-reported change in health were examined using the t-test for age and chi-square tests for all remaining variables. Age-adjusted and multivariable-adjusted logistic regression models were then specified to determine the association between each of the acculturation variables and change in health status. We created multiple models where each covariate was removed from the full model one at a time to examine its main effect and to test for confounding. Each covariate was found to be informative (considered as potential confounder) so final models included all covariates. A final model including all of the acculturation variables simultaneously was specified. Age at arrival in the U.S. was not included because it is a function of both age of interview and length of stay.

In examining change in health status, a central analytic challenge involves controlling for the effect of passage of calendar time or age. Health, particularly during midlife, is typically a negative function of age. However, since calendar time is indexed by time spent in the U.S., this variable reflects both the effects of aging and acculturation. Therefore, to estimate the net effect of time in the U.S., it was necessary to control for the effect of aging as well as developmental period in the lifecourse (i.e., calendar time). This was accomplished by stratifying by age group (i.e., < 31 years, 31-49 years, and 49 years or older) in order to control for developmental period, in addition to adjusting for chronological age in years. Results from both sets of analyses were not substantively different, however (results available upon request). Based on these comparisons, we concluded that analyses controlling for age were sufficient in determining the net effect of acculturation.

Potential moderation by race/ethnicity, gender, and health insurance status was examined for each of the primary independent variables by including the corresponding interaction terms. Selection of these variables was based on our prior hypothesis. In addition, we examined whether there may be differential associations between acculturation variables by country or region of origin in lieu of race/ethnicity. We hypothesized that these variables may be salient moderators, particularly for English language proficiency/use and dietary change variables, given that some countries or regions already have English as the primary language or have high rates of English fluency (e.g., some Caribbean countries, Canada, the United Kingdom) or are characterized by lifestyles that more closely resemble those of the U.S. All analyses applied sample weights and were conducted using SAS 9.2 (SAS Institute Inc, Cary, North Carolina).

## Results

The analytic sample contained primarily recent immigrants to the U.S. Twenty-six percent had resided in the U.S. for less than one year, and 35% for 1-5 years. In the overall sample, 43% was Hispanic, 30% was Asian, and the next largest group was White immigrants, followed by Black immigrants, and multiracial/other racial groups of immigrants. More than a third of respondents who had lived in the U.S. for ten years or less were Asian, while those who had lived in the U.S. for eleven or more years were predominantly Hispanic.

Bivariate analyses indicated that increasing age, and past and current smoking were associated with greater risk of reporting a worse change in health. Additional significant covariates were race/ethnicity, with Hispanic immigrants being most likely to report a worse change in health compared to those in other racial/ethnic groups; and marital status, with those who were divorced, widowed, or separated, being most likely to report a worse change in health. Significant acculturation variables associated with change in health status in bivariate analyses were length of stay, self-reported change in diet, and English language at work. Additional sociodemographic factors in the sample by change in health are presented in Table 1.

**Table 1:** Weighted descriptive characteristics of study participants by change in health status after moving to the United States (n=5,991).

***Variables***	**Change in Health Same/better**	**Change in Health**	**p value**
**N (%)**	**(n=5,410)**	**Worse (n=581)**	
**Age**	Mean=38.3SE=0.20	Mean=40.5SE=0.70	.0033
**Gender**			.2554
Male	2305 (42.6)	231 (39.8)	
Female	3105 (57.4)	350 (60.2)	
**Race/Ethnicity**			.0235
Asian	1661 (30.7)	147 (25.3)	
Black	477 (8.8)	29 (5.0)	
Hispanic	2280 (42.1)	292 (50.3)	
Multiracial/Other	67 (1.2)	8 (1.4)	
White	849 (15.7)	98 (16.9)	
Missing	76 (1.4)	7 (1.2)	
**Years of Education**			.1888
<12	2956 (54.6)	344 (59.2)	
12-16	1626 (30.1)	153 (26.3)	
>16	828 (15.3)	84 (14.5)	
**Length of Stay**			<.0001
<1 year	1525 (28.2)	53 (9.1)	
1-5 years	1931 (35.7)	175 (30.1)	
6-10 years	801 (14.8)	127 (21.9)	
11-15 years	736 (13.6)	140 (24.1)	
>15 years	417 (7.7)	86 (14.8)	
**Diet change**			<.0001
Completely the same (10)	955 (17.7)	72 (12.4)	
Very similar (6-9)	1662 (30.7)	158 (27.2)	
Somewhat different (5)	1005 (18.6)	92 (15.8)	
Very different (2-4)	734 (13.6)	103 (17.7)	
Completely different (1)	1054 (19.5)	156 (26.9)	
**English Speaking Ability**			.1155
Not Well	3031 (56.0)	302 (52.0)	
Well	2379 (44.0)	279 (48.0)	
**English Comprehension**			.0643
Not Well	2633 (48.7)	255 (43.9)	
Well	2777 (51.3)	326 (56.1)	
**Language at Home**			.3852
Not English	4404 (81.4)	462 (79.5)	
English	1006 (18.6)	119 (20.5)	
**Language at Work**			.0198
Not English	2772 (51.2)	267 (46.0)	
English	2489 (46.0)	306 (52.7)	
Missing	149 (2.8)	8 (1.4)	
**Language with Friends**			.7674
Not English	4089 (75.6)	443 (76.2)	
English	1321 (24.4)	138 (23.8)	
**Marital Status**			.0002
Never married	884 (16.3)	59 (10.2)	
Divorced/Widowed/Separated	423 (7.8)	59 (10.2)	
Cohabitating or Married	4103 (75.8)	463 (79.7)	
**BMI**			.0870
Underweight	234 (4.3)	20 (3.4)	
Normal	2632 (48.7)	247 (42.5)	
Overweight	1632 (30.2)	200 (34.4)	
Obese	656 (12.1)	81 (13.9)	
Missing	256 (4.7)	33 (5.7)	
**Exercise**			.0979
3x/week	805 (14.9)	65 (11.2)	
1-3x/week	3384 (62.6)	370 (63.7)	
None	1212 (22.4)	145 (25.0)	
Missing	9 (0.2)	1 (0.2)	
**Smoking status**			.0091
Never	4211 (77.8)	412 (70.9)	
Past	681 (12.6)	94 (16.2)	
Current	518 (9.6)	75 (12.9)	

Results from both age-adjusted and multivariable-adjusted models are presented in Table 2. Those who had been in the U.S. for 1-5 years, 6-10 years, 11-15 years, and 15 or more years, were all significantly more likely to report worse change in health since coming to the U.S. compared to those who had been in the U.S. for less than one year, both in age-adjusted and multivariate-adjusted models. In the multivariate-adjusted model, there was a graded positive association, with those who had been in the U.S. for 1-5 years having 2.69 times (95% CI: 1.87, 3.87), for 6-10 years having 5.24 times (95% CI: 3.50, 7.83), for 11-15 years having 6.20 times (95% CI: 4.13, 9.31), and for more than 15 years having 6.61 times (95% CI: 4.22, 10.36) the odds of reporting a worse change in health compared to those who had been in the U.S. for less than a year. This confirms our first hypothesis. Furthermore, those whose diets were “very different” or “completely different” since moving to the U.S. were about twice as likely to report worse change in health. Immigrants whose diet was very or completely different from their diet before immigration were more likely to have worse change in health (OR=1.98, 95% CI: 1.35, 2.90; OR=2.02, 95% CI: 1.40, 2.90, respectively) compared to people whose diet remained completely the same. This finding is consistent with our second hypothesis. Furthermore, in both age-adjusted and multivariable models, English proficiency variables became significantly associated with self-reported change in health, with those reporting greater ability to speak English (OR = 1.65, 95% CI = 1.30, 2.11) and those reporting better comprehension of English (OR = 1.65, 95% CI = 1.30, 2.10) being more likely to report a decline in health since moving to the U.S. compared to those who reported not being able to speak or comprehend English well, respectively. Those who reported speaking English at home or work were also more likely to report a worse change in health (OR=1.36, 95% CI: 1.01, 1.82; OR=1.75, 95% CI: 1.38, 2.22, respectively) (Table 2). However, speaking English with friends was not significantly associated with change in health. Most of these language related findings were consistent with our hypothesis.

**Table 2:** Associations between acculturation variables and change in health.

	**Change in Health**		
	**Age Adjusted Odds Ratio (CI**)†	Multivariate Adjusted Odds Ratio (CI)*	**Multivariate Adjusted Odds Ratio including all acculturation measures (CI)§**
**Length of Stay in U.S.**			
<1 yr	1.00	1.00	1.00
1-5 yrs	2.77 (1.93-3.97)	2.69 (1.87-3.87)	2.61 (1.78-3.81)
6-10 yrs	5.07 (3.45-7.45)	5.24 (3.50-7.83)	4.83 (3.15-7.42)
11-15 yrs	5.89 (4.04-8.59)	6.20 (4.13-9.31)	5.53 (3.61-8.48)
>15 yrs	6.05 (4.02-9.10)	6.61 (4.22-10.36)	5.90 (3.69-9.42)
**English Speaking Ability**			
Not Well	1.00	1.00	1.00
Well	1.32 (1.06-1.64)	1.65 (1.29-2.11)	1.11 (0.72-1.72)
**English Comprehension**			
Not Well	1.00	1.00	1.00
Well	1.39 (1.12-1.73)	1.65 (1.30-2.11)	1.03 (0.68-1.58)
**Language at Home**			
Not English	1.00	1.00	1.00
English	1.22 (0.92-1.61)	1.36 (1.01-1.82)	1.09 (0.78-1.53)
**Language at Work**			
Not English	1.00	1.00	1.00
English	1.43 (1.15-1.77)	1.75 (1.38-2.22)	1.23 (0.92-1.63)
**Language with Friends**			
Not English	1.00	1.00	1.00
English	1.04 (0.81-1.34)	0.92 (0.78-1.07)	0.82 (0.60-1.14)
**Diet Change**			
Completely the same (10)	1.00	1.00	1.00
Very similar (6-9)	1.32 (0.94-1.87)	1.36 (0.96-1.93)	1.25 (0.88-1.79)
Somewhat different (5)	1.28 (0.88-1.87)	1.36 (0.93-1.99)	1.18 (0.80-1.74)
Very different (2-4)	1.99 (1.36-2.91)	1.98 (1.35-2.90)	1.73 (1.17-2.57)
Completely different (1)	2.14 (1.50-3.04)	2.02 (1.40-2.90)	1.79 (1.23-2.60)

† Age adjusted model adjusted for age at interview only. Each acculturation measure is analyzed separately.

* Multivariate model adjusted for age at interview, gender, BMI categories, exercise, marital status, race/ethnicity, smoking, and years of education. Analyses weighted for sampling design of NIS. Each acculturation measure is analyzed separately.

§ Multivariate model adjusted for age at interview, gender, BMI categories, exercise, marital status, race/ethnicity, smoking, and years of education. Analyses weighted for sampling design of NIS. All acculturation measures are included in one model.

Interactions between acculturation variables and race/ethnicity and gender were not statistically significant. Health insurance was a significant effect modifier for associations between acculturation and change in health status. Among uninsured immigrants, there was a stronger association between increased length of stay and worse change in health status compared to insured counterparts. Detailed findings are published elsewhere [56]. Several additional models were specified including interactions between different combinations of countries/regions of origin and English language proficiency/use and dietary change variables. We expected differential associations with self-reported change in health status between participants from countries/regions of origin characterized by greater English proficiency or those more culturally resembling the U.S.; versus those where English is not a primary language or that are characterized by non-Western lifestyles. Contrary to what we hypothesized, these interactions were also not significant (results available upon request).

In the full model including all acculturation variables simultaneously, length of stay and self-reported change in diet remained significant predictors. However, none of the English language proficiency or use variables were significant.

## Discussion

Findings from our study provide mixed support that various indicators of acculturation among immigrants are associated with a decline in health. In the present study, acculturation (as measured by length of stay in the U.S., language skills/usage, and dietary change) was generally associated with elevated odds of reporting a negative change in health since moving to the U.S. This result is concordant with those of prior studies, which, albeit, have predominantly used current self-reported health status as the primary outcome [2,10,11,40,47]. In both age-adjusted and multivariable models including each of the acculturation variables separately, our study found significant associations between English proficiency variables and self-reported changes in health, with greater speaking ability and comprehension both being associated with greater odds of reporting a worse change in health. In addition, speaking English at home and at work were associated with greater odds of reporting a worse change in health compared to speaking a non-English language in these domains. However, in the full model including all of the acculturation variables, only length of stay and change in diet were significant, and none of the English language variables were significant. We examined whether the lack of significance of these variables was due to collinearity with other acculturation measures included in the model. Post-hoc analyses revealed acceptable inter-variable correlations between each of these measures.

There are several plausible reasons for the discrepancies in our findings. Firstly, English proficiency or use may not necessarily indicate assimilation to unhealthy U.S. norms or lifestyles. While for some immigrants, English language fluency may correspond with the adoption of poorer health behaviors, for others greater English proficiency may indicate integration and acceptance into U.S. culture more broadly. Indeed, some studies have suggested that discrimination based on language may be a particularly salient risk factor for poor health among immigrants [57]. Accordingly, those who do not speak or comprehend English may be more susceptible to language discrimination. Similarly, those who do not speak English in various domains may face exclusion from some dimensions of U.S. society. Although prior studies have suggested that English language proficiency and use may be associated with unhealthy assimilation, our results suggest that when taking into account additional aspects of the acculturative process, these factors may be less important when considering changes in the health of immigrants.

In contrast, we found that change in diet remained a significant predictor in our final model. Interestingly, those who reported more change in one’s diet were also more likely to have stayed in the U.S. longer. This demonstrates that dietary change is a very good measure for acculturation. Our results specifically point to dietary change as a potential mechanism through which acculturation may lead to worsening health among immigrants. Poor health behaviors may be acquired upon immigration to the U.S., such as those around diet and sedentary lifestyle, as supported by other studies showing a higher prevalence of overweight and obesity in acculturated immigrants [58]. Diet change could also be a proxy for assimilation to a particular environment (such as not having access to ethnic foods familiar from home). These may partially explain our findings.

In addition, length of stay was also a significant predictor in our final model even after adjusting for age which controls for passage of calendar time. One possible reason that length of stay remained strongly associated with change in health is that duration in the U.S. may be a particularly robust marker of unhealthy assimilation. Although acculturation may be associated with socioeconomic advantages, it may have detrimental effects on health [33]. While some researchers have posited that acculturation among immigrants may result in access to healthcare services not available in their countries of origin [59], or may discourage health-damaging behaviors that may be culturally normative (e.g., smoking, physical inactivity, lack of preventive screening) [60-63], our findings are concordant with those of prior studies suggesting that length of stay, when interpreted as a marker of acculturation, results in a net detrimental effect on health. An alternative explanation of this finding is that length of stay may reflect greater exposure to psychosocial hazards commonly experienced by immigrants. Other studies have suggested that longer duration in the U.S. may be associated with greater exposure to various sources of stress, including acculturative stressors arising from adjustment to a new culture, the experience of racial discrimination, as well as language barriers [64-71]. Additionally, length of stay could reflect change in how people rate their health.

There are several caveats to our findings to be noted. First, the sample consists only of immigrants who were granted legal permanent residency between May and November 2003, which may exclude longtime U.S. dwellers. In fact, 26% of our sample lived in the U.S. for less than a year, and 35% had lived in the U.S. for 1-5 years. Also, a group of people that obtains permanent residency after less than one year may be a highly select group, and they may be fundamentally different in some characteristics from individuals who obtain permanent residency after a longer duration. This feature of the sampling design may limit generalizability of our findings to all U.S. immigrants. This study also does not include undocumented or temporary residents. Although change in health status may provide relatively new and meaningful information to the literature, this question may entail a potential problem of not accurate recall of their health status before immigration, especially among those who stayed in U.S. longer. Although the use of self-reported change in health as our primary outcome may appear less rigorous than clinical health outcomes, prior studies on self-reported measures of overall health have consistently shown it to be a robust indicator of current health as well as mortality, even after the inclusion of covariates known to predict mortality [72]. For example, using longitudinal data from more than 700,000 participants in the NHIS, those who reported their health as fair or poor had at least a two-fold risk of subsequent mortality (using data from the National Death Index), and this relationship was true among all racial groups including Hispanics, Blacks and Asians/Pacific Islanders [73]. Accordingly, self-reported change in health may be a reliable and valid measure, and also have implications for actual health and mortality. Change in diet was measured using one item in the survey, and therefore, it was not able to capture a very complex nature of dietary behavior such as changes in consumption of fat, fast food, etc. Also, reasons for changing diet were not available in the dataset. Additionally, the New Immigrant Survey did not collect information on physical environment such as pollution, water, or food, so we were not able to assess influence of physical environment on health of participants.

Our study is characterized by several strengths that make it an important contribution to the existing literature. Firstly, the use of change in health status since moving to the U.S. is an important strength of this study. Change in health may more accurately represent the impact of immigration compared to the use of self-reported current health because respondents’ reference point is their own health prior to immigrating. We were also able to adjust for several important health behaviors and attributes such as smoking, physical activity, and body mass index in our study. Our findings suggest that acculturation may have an effect on health above and beyond these potential mechanisms. Secondly, we included multiple measures of acculturation in this study (length of stay; English speaking and comprehension skill; speaking English or native language with family, friends, and coworkers; and change in diet since immigration). As these diverse measures capture multiple aspects of acculturation, our study presents a richer description of the dynamics involved in immigration. The use of single measures of acculturation may not capture the various facets of acculturation. For example, a long-time immigrant residing exclusively in an isolated ethnic enclave may not be as acculturated as a more recent immigrant living in a racially or ethnically integrated neighborhood. Furthermore, by considering these multiple indicators together, we were able to tease out which acculturation variables were more strongly associated with change in health status when they were considered simultaneously in one model. Thirdly, we examined a large sample of immigrants representing at least 21 countries from six continents. These immigrants reside across all regions of the U.S, representing all of the top 85 Metropolitan Statistical Areas. Being more representative of the entire U.S. immigrant population, results of this study may be more generalizable to the national level compared to those which have focused on specific national origin groups or those in specific geographic areas.

These results lend support to the hypothesis that acculturation, and particularly dietary change, is associated with a declines in health among immigrants. Although few would contest the benefits of integrating into the host society – typically manifested through language acquisition, educational attainment, occupational status, homeownership, wealth, and political participation – this acculturative process seems to have deleterious effects on immigrant health. Further, the socioeconomic gains that are typically associated with positive health outcomes are somewhat negated by this acculturative process. Our study also suggests that English language proficiency and use, though a typically studied proxy for acculturation, may not necessarily constitute a risk factor for poor health among immigrants when controlling for other aspects of acculturation. Duration of stay, however, may be a particularly relevant marker of assimilation to less healthy U.S. lifestyles or exposure to psychosocial stressors typically experienced by immigrants, such as racial, language, and anti-immigrant discrimination. Future research incorporating a longitudinal study design focusing on changes in health and multidimensional aspects of the context of acculturation is warranted. In addition, studies that include both physical and mental health outcomes may present a more comprehensive picture of the relationship between acculturation and health among immigrants. Both an understanding of the factors that help immigrants retain their positive health profiles as well as further disentanglement of the structural and psychosocial stressors that contribute to health declines is needed going forward.
